# Traditional Chinese Medicine Based Acupoint Application for Asthma Treatment in Children: A Meta-Analysis and Systematic Review

**DOI:** 10.1155/2022/7500056

**Published:** 2022-09-26

**Authors:** Yijie Wang, Tingting Guo, Fushuang Yang, Yongjun Li, Lujia Liu, Kexin Lin, Zhijun Li, Youpeng Wang

**Affiliations:** ^1^Heilongjiang University of Chinese Medicine, Harbin 150040, China; ^2^Changchun University of Chinese Medicine, Changchun 130117, China; ^3^The Second Affiliated Hospital of Heilongjiang University of Chinese Medicine, Harbin 150009, China

## Abstract

**Objective:**

By conducting a systematic review of the efficacy of acupoint application on children with asthma.

**Methods:**

We searched Chinese databases (CNKI, VIP, and Wanfang) and English databases (PubMed, Embase, and Cochrane Library) for studies from the establishment of the database to October 2021. The included literature studies were randomized control studies investigating the treatment of asthma in children by acupoint application. The primary outcomes included the cure rate, the resolution time of cough, and the resolution time of wheezing. The secondary outcomes included pulmonary function and interleukins. Stata 15 and RevMan 5.4 were used to analyze the extracted data.

**Results:**

A total of 24 related studies were included containing 2716 cases. The meta-analysis showed that TCM group was superior to control group in terms of cure rate, pulmonary function (FEV1), and resolution time of wheezing in children with asthma [RR = 1.26,95% (1.21,1.31), *P* < 0.05; SMD = 0.81, 95%CI (0.05,1.56), *P* < 0.05; WMD = −1.40, 95%CI (−1.75, −1.05), *P* < 0.05].

**Conclusions:**

The present study shows that acupoint application is an effective treatment for children with asthma in China, especially in alleviating wheezing and improving quality of life.

## 1. Introduction

Asthma is a chronic and refractory disease that affects the quality of human life globally. This chronic inflammation is mainly related to airway hyper-responsiveness and reversible airflow limitation, which causes symptoms such as recurrent wheezing, shortness of breath, chest tightness, and cough [1]. In recent years, the incidence of asthma was increasing year by year. At present, there are about 334 million children with asthma in the world and 30 million children with asthma in China [2, 3]. Respiratory symptoms in children aged 5 to 16 years lack specificity, and they could develop asthma-like symptoms which may be caused by respiratory virus infection or prolonged disease course [4]. This results in overdiagnosis and abuse of adrenal cortical hormones (hormones), which make children and their families bear unnecessary costs and adverse reactions [5]; traditional Chinese medicine has a good clinical effect on children with asthma with low recurrence rate and side effects.

Asthma is a refractory disease with high rates of recurrence [6]. Therefore, the treatment principle of this disease in clinical practice basically aims to control the disease progression. Inhaled glucocorticoids, long-acting*β*2-receptor agonists (LABA), and leukotriene receptor antagonists are the main controller medications. Short-acting*β*2 receptor agonists (SABA) and inhaled anticholinergic drugs are the main relief drugs [7]. Acupoint application of traditional Chinese medicine has a long history. Acupoint application treatment is based on syndrome differentiation and treatment; transdermal drug delivery can avoid the first pass effect of gastrointestinal digestive fluid and the liver and also avoid the “peak-valley phenomenon”. In addition, the interlayer of skin tissue structure has storage capacity, which can make the blood concentration curve of drugs entering human tissues gentle and lasting. Previous studies reported that acupoint application could be used to treat childhood bronchial asthma, and the effective rate could reach 100% [8]. According to the theory of acupoint application, the mechanisms of asthma include acute airway obstruction and inversion of lung Qi which are mainly caused by long-term phlegm retention in the lungs and further aggravated by emotions, diet, fatigue, and physical weakness. Some studies believed that the pathogenesis of childhood bronchial asthma is retaining phlegm, which is directly related with the dysfunction of the liver, spleen, and kidneys. Exogenous lung wind, improper diet, and blockage of chest yang can contribute to asthma [9, 10]. However, the efficacy of acupoint application of traditional Chinese medicine in the treatment of childhood asthma is still unclear. Thus, a meta-analysis was conducted to compare the efficacy of acupoint application in the treatment of childhood asthma.

## 2. Materials and Methods

This meta-analysis was conducted in accordance with the Preferred Reporting Items for Systematic Reviews and meta-analysis (PRISMA) statement [11]. Scientific databases (PubMed, Embase, Web of Science, Cochrane Library, CBM, CNKI, and Wanfang) were comprehensively searched to identify relevant literature studies without language restriction. Relevant keywords, medical terms, and titles include acupoint application, children, asthma, and randomized controlled trials. The search results included original research papers published in online journals as of October 29, 2021, Specific search method, Supplementary material 1.

### 2.1. Inclusion and Exclusion Criteria

According to the aims of the study, the inclusion criteria were as follows: (1) the included population should meet the diagnostic criteria for asthma, (2) age <15 years old, (3) acupoint application intervention is the main therapeutic approach, (4) randomized controlled trials, and (5) complete original data.

Exclusion criteria were as follows: (1) conference abstracts and systematic reviews, (2) repeated publications, (3) animal experiments or nonclinical experiments, (4) articles with unreasonable experimental design, and (5) full text was not available.

### 2.2. Data Extraction

The following data were extracted from each eligible study: first author, country, subjects, number of participants, sex, age, intervention, comparator, treatment stage, treatment duration, follow-up time, lung function, cure rate, the resolution time of wheezing, serum IgE, and other related data. To ensure the quality of the meta-analysis, all eligible articles were independently reviewed and cross-checked by 2 researchers according to standardized methods. If there was any dissent, another reviewer was consulted. A consensus was reached on the selection of the final included studies.

### 2.3. Risk of Bias Assessment

Cochrane risk of bias tool was used to evaluate the risk of bias of each studies containing RCT and the following factors were taken into account: random sequence generation, allocation concealment, blinding of participants and researchers, blinding of outcome assessments, incomplete outcome data, selective reports of outcomes, and other sources of bias. The risk of bias in each aspect was scored as low, high, or unclear risk [12].

### 2.4. Statistical Analysis

Stata/SE12.0 software was used in this meta-analysis. The pooled enumeration data were expressed as relative risk (RR) and 95% confidence interval (CI). The pooled continuous variables were expressed as mean standard deviation (MD) and 95% CI operation. *P* < 0.05 was used as the standard to determine the difference to be statistically significant. *Q*-test (*P-*value) and chi-square test (I2) were used to determine the heterogeneity. The heterogeneity was considered not significant if *P* ≥ 0.1 and I2 ≤ 50%, and the fixed-effects model was used to pool the data. Otherwise, the random-effects model was used to pool the data. The subgroup analysis was used to determine the source of the heterogeneity. Egger's test was performed to evaluate the publication bias, and *P* > 0.05 indicated that there was no publication bias; otherwise, publication bias existed.

## 3. Results

### 3.1. Literature Search and Screening

A total of 895 articles were initially retrieved. 563 articles were selected after removing duplicated publication. 464 articles were removed by reading the title and abstract. After reading the full text, 75 articles were removed due to incomplete results, unavailable data, and low quality of the literature, and 24 articles were finally involved in this analysis [13–34] with a total of 2716 patients. The flow chart of literature search is shown in Figure 1.

### 3.2. Basic Characteristics and Quality Evaluation of the Included Literature

The 24 literature studies included in this analysis were all randomized controlled studies published in Chinese. A total of 2716 subjects were included, among which 1384 subjects were in the experimental group and 1332 in the control group. The detailed characteristics of the literature are shown in Table 1. The plot for risk of bias is shown in Figure 2.

### 3.3. Meta-Analysis Results

#### 3.3.1. Cure Rate

There were 18 studies [13–17, 19–23, 26, 27, 29–32, 35, 36] mentioning the cure rate of the two groups which was expressed as dichotomous variables. The treatment stage was used for subgroup analysis. The fixed-effects model was employed (I2 = 48.1%, *P* = 0.012), and the pooled results showed that there was a statistically significant difference between the two groups [RR = 1.26, 95% (1.21, 1.31), *P* < 0.05]. The meta-analysis results presented that the effect of acupoint application was significantly superior to that of the control group in treating childhood asthma (Figure 3(a)).

A funnel plot was used to directly visualize publication bias, and Egger's and Begg's tests were used to analyze the funnel plot. The results of Egger's and Begg's test showed no significant difference (*P* < 0.05). Additionally, the results of sensitivity analysis showed that after excluding the study one by one, there was no significant change in effect size (Figures 3(b), 3)(c).

#### 3.3.2. Pulmonary Function (FEV1)

In the included articles, 8 studies [15–17, 22, 24, 28, 29, 33] mentioned FEV1-related indicators, which were presented as continuous variables. The random-effects model (I2 = 96.7%, *P* = 0) was used to pool the effect size, and the pooled results showed that the difference between the two groups was statistically significant [SMD = 0.81, 95%CI (0.05, 1.56), *P* < 0.05]. The meta-analysis results presented that the effect of acupoint application was significantly superior to that of the control group in improving pulmonary function (Figure 4(a)).

A funnel plot was used to directly visualize publication bias, and Egger 's and Begg 's tests were used to analyze the funnel plot. The results of Egger 's and Begg 's test showed no significant difference (*P* < 0.05). Additionally, the results of sensitivity analysis showed that after excluding the study one by one, there was no significant change in effect size (Figures 4(b), 4(c)).

### 3.4. Function (FEV1)

#### 3.4.1. The Resolution Time of Wheezing

A total of 4 papers [13,22,28,33] reported the resolution time of wheezing, which was presented as a continuous variable. The random-effects model (I2 = 85.8%, *P* = 0) was used to pool the effect size. The pooled results showed that the difference between the two groups was statistically significant [WMD = −1.40, 95%CI (−1.75, −1.05), *P* < 0.05]. The meta-analysis results presented that the effect of acupoint application was significantly superior to that of the control group in improving asthma symptoms in children (Figure 5(a)). Sensitivity analysis showed that there was no significant change in effect size after removing the studies one by one (Figure 5(b)).

#### 3.4.2. Serum IgE Level

A total of 4 studies [13, 17, 26, 35] reported serum IgE level which was expressed as continuous variables. The random-effects model (I 2 = 99.1%, *P* = 0) was used to pool the effect size. The pooled results showed that the difference between the two groups was not statistically significant [SMD = 1.39, 95%CI (−0.65, 3.44), *P* < 0.05]. The meta-analysis results demonstrated that there was no significant difference between the experimental group and the control group in the IgE level (Figure 6).

#### 3.4.3. Occurrence of Asthma

A total of 4 [14, 31, 35, 37] studies reported the occurrence of asthma which were expressed as continuous variables. The random-effects model (I 2 = 98.2%, *P* = 0) was used to pool the effect size. The pooled results showed that the difference between the two groups was not statistically significant [ SMD = −0.89, (−2.82, 1.04), *P* > 0.05]. The meta-analysis results demonstrated that there was no significant difference between the experimental group and the control group in the occurrence of asthma (Figure 7).

## 4. Discussion

With the improvement of medical conditions, increasing attention has been paid to the prevention and treatment of asthma. However, due to air pollution, changes in living and diet habits, and other factors [38], the incidence of childhood asthma has been increased. From the perspective of TCM, asthma belongs to the category of “wheezing disease” as termed by TCM. This concept was first mentioned in the “Huangdi Neijing”. Wheezing disease is recurrent due to the failure in completely removing the etiological factor, subsequently aggravated by repeated exposure to exogenous pathogens [39]. Traditional Chinese medicine classifies asthma as “wind-cough” and “wheezing cough,” and the treatment scheme adopts the principle of syndrome differentiation and treatment, treating both inside and outside. Li Yue Parallel Prose once said, “The reason of external governance is the reason of internal governance. Though it is treated externally, nothing can be treated internally.” External treatment and internal treatment can complement and coordinate each other. Acupoint application has a long history in the external treatment of asthma. It can directly act on specific acupoints of the human body, and its multiple effects such as comprehensive drugs, acupoints, and meridians will direct the efficacy of the disease [39]. Based on the comprehensive analysis of the included literature studies, most of the basic drugs used for acupoint application were Chinese mustard seed, Asarum, Euphorbia kansui, and Rhizoma corydalis. White mustard has the function of warming lung and reducing phlegm. Relevant studies show that the efficacy of white mustard in adhesive can quickly penetrate into the skin and release stably [40]. Asarum pungent and warm, return to the heart, lung, and kidney meridian, has the effect of warming lung and hua Yin, etc. Asarum volatile oil can inhibit the release of inflammatory mediators, reduce histamine content, and fight against histamine or prostaglandin E caused by increased capillary permeability. Euphorbia kansui bitter cold, belongs to the lung, kidney, and spleen meridian, has the effect of purging water by drinking. Rhizoma corydalis tastes hard, warm, goes to the liver and stomach meridian, with qi, pain, blood circulation, and blood stasis [41]. The combination of the four herbs has the effect of relieving phlegm and benefiting qi, warming lung, and relieving cough. Acupoints are applied at the locations of lung acupoints, ding asthma acupoints, spleen deficiency, kidney deficiency, etc. The back acupoints are closely related to the sympathetic nerve. Stimulating acupoints can excite the sympathetic nerve, reduce the vagus nerve tension, and have the effect of relieving spasm and relieving cough [42].

The external therapy in acupoint application is an important approach to treat childhood asthma [43]. This therapy is easy to use, simple to operate, and good in compliance, showing a definite and rapid effect. Treatment is mainly based on acupoint application, pediatric massage, acupuncture, nasal drip of acupoint application, and fumigation and washing by using acupoint application. Among them, acupoint application is a common treatment method in pediatrics. Acupoint application can exert multiple effects in the treatment of asthma. The drug can not only be absorbed through the skin but can also promote the relaxation of bronchial smooth muscle, and thus dilate the bronchus and improve the symptoms of airway spasm. Meanwhile, through the special physiological amplification effect of the meridian points, it can exert anti-inflammatory effects, adjust the immune function of the body, improve blood circulation, and regulate the functions of the nerves, body fluids, and endocrine system, etc. Xunbin et al. [44] reported 111 cases and used acupoint application (Baijizi, Corydalis, Asarum, cinnamon, ginger juice, and starch) to conduct acupoint application on the specific points (Shuangfeishu, Shuangxinshu, Shuanggeshu, Shuangzusanli, Shuangfengmen, ShuangjueYinshu, Shuanggeshu, and Shuangpishu points). The results showed that the treatment was remarkably effective in 50 cases, effective in 7 cases, and ineffective in 2 cases, with a total effective rate of 96.1%. Yang Yafeng [45] treated childhood bronchial asthma by acupoint application, and the total effective rate was 92.5% after 1 year. It showed that the adjuvant therapy of acupoint application was also rather important in acute asthma attack. For children treated with Western medicine alone, the effective rate was 84.5%. The effective rate reached 97.9% after a combined use with acupoint application treatment. Acupoint application exerts a satisfactory auxiliary effect on the treatment of childhood bronchial asthma, which improves the clinical efficacy. This method is easy to operate in clinical practice, and it is safe and reliable for children to use without pain.

This study had several limitations. First, although we attempted to address heterogeneity through subgroup and sensitivity analyses, the heterogeneity in statistics and clinical data might raise doubts about the validity of this study. The heterogeneity of the study population made it challenging to prove that the results were meaningful. Second, the sample size was small, and the occurrence of asthma was low in many included studies with low quality. Third, the source of the research object is single. Thus, the uncertainty in the analysis was increased. The RCT methods in the included studies were generally poor since most risk items were unclear, especially the allocation concealment, blindness, and selective outcome reporting. This limitation might reduce the credibility of our conclusions.

## 5. Conclusion

The present study shows that acupoint application is an effective treatment for children with asthma in China, especially in alleviating wheezing and improving quality of life. Due to the limitations of the study, further research should be conducted in the future with rigorous design, large sample size, sham/placebo control or blank/waiting control, and accurate report to support the evidence of acupoint application treatment in childhood asthma. Furthermore, since all studies were conducted in China, further studies in other countries are necessary to improve the applicability and generalizability of the results.

## Figures and Tables

**Figure 1:** Results of literature screening and the process.

**Figure 2:** Risk of bias summary and graph.

**Figure 3:** Forest plot, funnel plot, and sensitivity analysis of meta-analysis on cure rate.

**Figure 4:** Forest plot, funnel plot, and sensitivity analysis of meta-analysis on pulmonary function (FEV1).

**Figure 5:** Forest plot and sensitivity analysis of meta-analysis on the resolution time of wheezing.

**Figure 6:** Forest plot of meta-analysis on serum IgE level.

**Figure 7:** Forest plot of meta-analysis on the occurrence of asthma.

**Table 1:** Basic information of the included literature.

Number	Year	Author	Journal	Study type	Country	Intervention		Case		Age(mean ± sd)		Gender (male/female)		Stage	Period of treatment	Follow-uptime
						Treatment group	Control group	Treatment group	Control group	Treatment group (year)	Control group (year)	Treatment group	Control group			
1	2009 [19]	Guo Juzhen	Journal of Sichuan of Acupoint Application	RCT	China	Inhalation of pumice aerosol, combined with acupoint application acupoint external application treatment	Just inhale pumice aerosol	40	32	—	—	23/17	18/14	—	30 days	3 to 6 months

2	2009 [20]	HE Wei	Chin Pediatr Integr Tradit West Med	RCT	China	Based on the treatment of relieving spasmolysis and relieving asthma, intermediate frequency drugs were added to the acupoint for treatment	Treatment of spasmolysis and asthma	60	60	—	—	40/20	46/14	Attack	3 days	—

3	2010 [21]	HU Aie	China Modern Doctor	RCT	China	The aerosol inhalation of Pulmicort in acute episode of asthma and the Chinese herbal acupoint application in its remission period were given to the treatment group	The aerosol inhalation of Pulmicort in acute episode of asthma was given to the control group	50	50	2.4	1.9	30/20	31/19	Duration and remission	3 years	—

4	2011 [26]	SHI Danmei	Clinical Journal of Chinese Medicine	RCT	China	Inhalation budesonide suspension + albuterol atomization solution + inhalation ipratropium bromide atomization, plus Chinese medicine acupoint application	Inhalation budesonide suspension + albuterol atomization solution + ipratropium bromide atomization solution for inhalation treatment	154	150	—	—	73/81	67/83	-	7 days	—

5	2010 [25]	Shi Pinying	Journal of Acupoint Application	RCT	China	On the basis of inhaling seretide for 6 months, Wu's blistering plaster for acupoint application was applied in dog-days	Treated with seretide inhalation 50 *μ*g/100*μ*	40	40	7.9 ± 1.5	8.2 ± 1.9	23/17	24/16	In remission stage	6 months	—

6	2011 [32]	Zhang Xiuying	J. Pediatrics of TCM	RCT	China	Fu Jiu sticking therapy was administered in combination with beclomethasone dipropionate aerosol or budesonide inhalation powder	Treated with beclomethasone dipropionate aerosol or budesonide inhalation powder	60	60	—	—	38/22	39/21	In remission stage	3 years	—

7	2012 [15]	Deng Yuping	Hubei Journal of TCM Aug	RCT	China	On the basis of the treatment with inhalation of seretide powder, the treatment of winter disease in summer was added. On the first day of Tou Fu, Erfu, and Sanfu in summer every year, Sanfu acupoint application of cough and asthma was given	Treatment with inhalation seretide powder was given	80	80	7.59 ± 3.31	7.86 ± 2.95	48/32	45/35	In remission stage	1 year	—-

8	2012 [24]	Luo Jing-yan	Tianjin Med J	RCT	China	According to GINA regimen, inhaled glucocorticoid-based stepwise treatment was given, and inhaled budesonide aerosol was selected, on this basis, siji ointment was applied at point 2	Inhaled glucocorticoid-based step therapy was administered according to the GINA protocol, using budesonide aerosol inhalation	75	51	6.5 ± 1.3	6.4 ± 1.4	43/32	27/24	Duration	6 weeks	6 months

9	2012 [25]	Luo Jing-yan	Tianjin Journal of Acupoint Application	RCT	China	Inhaled glucocorticoid-based step therapy was administered according to the GINA protocol, using budesonide aerosol inhalation	Inhaled glucocorticoid-based step therapy was administered according to the GINA protocol, using budesonide aerosol inhalation	56	42	8.74 ± 1.64	8.61 ± 1.57	33/23	25/17	Duration	Once every 7=10 days, 6 times as a course of treatment	6 months

10	2012 [29]	Wu Fang	China Journal of Chinese Materia Medica	RCT	China	Xiaochuangao acupoint paste combined with fluticasone propionate aerosol	Inhale fluticasone propionate aerosol	30	30	7.6 ± 2.4	7.9 ± 2.5	15/15	16/14	In remission stage	1 year	1 year

11	2015 [34]	Zhao Juan	Clinical Journal of Acupoint Application	RCT	China	In addition to the routine use of glucocorticoid inhalation, observation group (20 cases) dog days into the volt is given selfmade acupoint application paste acupoint sticking	Used conventional glucocorticoid inhalation therapy	20	20	—	—	—	—	In remission stage	1 year	1 year

12	2016 [17]	Fang Junmei		RCT	China	On the basis of inhaling budesonide at less than 5 years old and inhaling sulide at more than 5 years old, combined with point mounting method during the dog and coldest days	Younger than 5 years, inhaled budesonide, older than 5 years, inhaled seretide	160	160	2.5-12	1.5-13	92/68	89/71	Duration	1 year	—

13	2017 [18]	Gu Hongdan	Chinese Archives of acupoint application	RCT	China	Treated with Xiao Chuan paste acupoint application combined with fluticasone propionate aerosol	Inhale fluticasone propionate aerosol	50	50	9.73 ± 2.42	9.65 ± 2.52	28/22	26/24	In remission stage	1 year	1 year

14	2017 [23]	Li Guiying	Journal of Clinic Nursing's practicality	RCT	China	Albuterol atomized inhalation combined with magnetic patch (acupoint application therapy) treatment	Treated with aerosol inhalation of salbutamol	40	40	—	—	—	—	—	30 days	—

15	2011 [25]	Shen Yi-yun	Guiding Journal of Acupoint Application and Pharmacology	RCT	China	On the basis of atomizing inhalation of Pulmicort, Bricanyl, and ipratropium bromide, acupoint sticking therapy with clearing heat stick combined with iontophoresis technology was given	Treated with Pulmicort, Bricanyl, and ipratropium bromide inhalation	60	60	6.53 ± 3.34	6.53 ± 2.09	31/29	28/32	Attack	5 days	—

16	2017 [28]	Shu Yifang	Journal of Clinical Medicine in Practice	RCT	China	Treated with the combination of budesonide and acupoint application with Chinese herbal medicine	Treated with budesonide atomization inhalation	40	40	9.1 ± 0.7	9.5 ± 0.5	19/21	24/16	—	36 days	—

17	2017 [35]	Zhou Fang	Chinese Journal of Traditional Medical Science and Technology	RCT	China	On the basis of inhaling pumice aerosol, wenyang Qucold paste was applied at summer acupoint	Give pumice aerosol inhalation	44	42	—	—	—	—	In remission stage	Three volts a course of treatment	—

18	2018 [36]	Zhao Meili	Guangxi Journal of Acupoint Application	RCT	China	Fluticasone propionate aerosol combined with acupoint application treatment, “relieving asthma cough external application powder”	Inhale fluticasone propionate aerosol	50	50	10.23 ± 2.85	9.66 ± 2.93	25/25	20/30	In remission stage	The experimental group was treated for 4 weeks as a course of treatment, the control group was treated for 10 days as a course of treatment, and the control group was treated with 4 times of application as a course of treatment	—

19	2020 [16]	Fan Xiaoni	Contemporary Medical Symposium	RCT	China	Salbutamol combined with acupoint stimulation was used for treatment	Treated with aerosol inhalation of salbutamol	40	40	4.57 ± 0.45	4.85 ± 0.46	23/17	22/18	Attack	2 weeks	—

20	2020 [33]	Zhao Baoling	Inner Mongolia Med J	RCT	China	Budesonide inhalation atomization treatment combined with “winter disease treatment in summer” three Fu stickers	Treated with budesonide atomization inhalation	49	49	9.33 ± 1.84	9.19 ± 1.73	24/25	26/23	—	36 days	—

21	2021 [22]	Le Lijun	Journal of Hubei Polytechnic University	RCT	China	Treated with acupoint application combined with budesonide atomization inhalation and symptomatic treatment	Treated with budesonide atomization inhalation	48	48	4.74 ± 2.87	4.34 ± 2.18	25/23	23/25	—	A course of treatment was given every week for 2 weeks	—

22	2021 [30]	Xie Jianling	Selfcare	RCT	China	On the basis of drug atomization inhalation treatment, acupoint application of “Shuji Point” was given	Treated with drug atomization inhalation	50	50	6.5 ± 3.1	6.1 ± 3.0	26/24	28/22	Duration	3 weeks	—

23	2021 [31]	Yang Dongyan	Practical Clinical Journal of Integrated Traditional Chinese and Western Medicine	RCT	China	Routine inhalation of budesonide aerosol treatment and Chinese medicine treatment of winter disease summer acupoint application	Treated with budesonide atomization inhalation	38	38	7.28 ± 0.49	7.30 ± 0.51	—	—	In remission stage	3 months	—

24	2015 [14]	Chen Yan	Today Nurse	RCT	China	Add acupoint application on the basis of Singulair or sulfone sprays	Treatment was given with Singulair or sulfone sprays	50	50	—	—	27/23	24/26	In remission stage	3 summer	—

## Data Availability

The data that support the findings of this study are available from the corresponding author upon reasonable request.

## Supplementary Materials

Supplementary Materials 1. PRISMA_2020_checklist was uploaded as a supplementary file. 2. Search strategy was uploaded as a supplementary file. .
